The article "Efficacy of Cetuximab in Nasopharyngeal Carcinoma Patients Receiving Concurrent Cisplatin-Radiotherapy: A Meta-Analysis" was retracted in 2023. Reasons: unreliable results or conclusions; concerns about the data; concerns about the peer review; concerns about the citations.

# Efficacy of Cetuximab in Nasopharyngeal Carcinoma Patients Receiving Concurrent Cisplatin-Radiotherapy: A Meta-Analysis

**DOI:** 10.1155/2022/5145549

**Published:** 2022-08-24

**Authors:** Lin Wang, Dianjun Liu, Deyou Wei

**Affiliations:** ^1^Department of Pharmacy, Yantaishan Hospital, Yantai, Shandong 264001, China; ^2^Department of Pharmacy, Yantai Hospital of Traditional Chinese Medicine, Yantai, Shandong 264001, China; ^3^Department of Otolaryngology, Yantai Hospital of Traditional Chinese Medicine, Yantai, Shandong 264001, China

## Abstract

**Background:**

Nasopharyngeal carcinoma (NPC) is a malignant neoplasm of the nasopharyngeal epithelium. Concurrent chemoradiotherapy has been established as a standard treatment for locoregional NPC, and cisplatin is a common agent in NPC treatment. Cetuximab is a monoclonal antibody against epidermal growth factor receptor. This meta-analysis was performed to evaluate the curative effectiveness and survival outcomes of cetuximab in NPC patients who received concurrent cisplatin-radiotherapy.

**Methods:**

PubMed, Cochrane Library, EMBASE, China National Knowledge Infrastructure (CNKI), Wan Fang, and China Biology Medicine disc (CBM) were used to search publications studying on concurrent chemoradiotherapy and/or cetuximab in NPC. The qualities of included RCTs were assessed by the Newcastle-Ottawa Scale. STATA 14.0 was used to conduct the statistical analysis.

**Results:**

In total, 17 trials with 2066 patients were included in this meta-analysis. The results from this study show that cetuximab improved the therapy efficacy in NPC patients who received concurrent cisplatin-radiotherapy. Cetuximab cotreatment improved the complete response (RR = 1.92, 95% CI [1.61, 2.30]), and reduced stable disease (RR = 0.67, 95% CI [0.51, 0.88]) as well as progression disease (RR = 0.24, 95% CI [0.15, 0.40]). Besides, it also improved the overall survival (RR = 1.10, 95% CI [1.02, 1.18]), disease-free survival (RR = 1.09, 95% CI [1.03, 1.15]), metastasis-free survival (RR = 1.06, 95% CI [1.01, 1.11]), and relapse-free survival (RR = 1.04, 95% CI [1.01, 1.07]) in NPC patients.

**Conclusions:**

Cetuximab could improve the curative efficacy and survival outcomes of NPC patients who underwent concurrent cisplatin-radiotherapy. However, all the trials included were conducted in China; thus, the quality of the trials in this study remains doubtful. More high-quality RCTs should be included in further relevant studies.

## 1. Introduction

Nasopharyngeal carcinoma (NPC) is an epithelial carcinoma associated with the nasopharyngeal mucosa, and it is closely associated with Epstein-Barr virus (EBV). When comparing with other cancers, NPC is quite uncommon. In 2018, there were approximately 129,000 new cases of NPC, which represents only 0.7% of all cancer types diagnosed [1]. NPC occurs frequently in the south of China and Southeast Asian countries, and men have a higher incidence of NPC than women [2].

The article "Efficacy of Cetuximab in Nasopharyngeal Carcinoma Patients Receiving Concurrent Cisplatin-Radiotherapy: A Meta-Analysis" was retracted in 2023. Reasons: unreliable results or conclusions; concerns about the data; concerns about the peer review; concerns about the citations.

Advances in radiation therapy technology and concomitant chemotherapy have led to improvements in the management of NPC [3]. In comparison to traditional 2D or 3D radiation therapy, intensity-modulated radiotherapy (IMRT) is ideally suited to the target area of the tumor, as it can deliver a high dose of radiation to NPC while protecting adjacent tissues and reduce adverse effects including neurotoxicity and dysphagia [4, 5]. NPC is a chemotherapy-sensitive disease. Combined agents, particularly cisplatin-based regimes, are highly effective in the treatment of NPC [6].

In the epoch of traditional 2D radiation therapy, studies have shown that, compared to radiation alone, simultaneous chemoradiation may significantly improve the 5-year overall survival and progression-free survival in patients with stage II NPC [7]. However, other studies have shown the opposite. Al-Sarraf et al. and Lee et al. indicated that the concomitant chemoradiation group was not greater than those in the IMRT group in patients with NPC. Studies have confirmed that concomitant chemoradiation therapy accompanied by adjuvant chemotherapy or not could lead to better outcomes than radiotherapy alone in stage III-IV locoregionally NPC [8, 9]. On the contrary, neither adjuvant chemotherapy nor induction chemotherapy could improve the survival outcomes of radiation therapy; thus, concurrent chemoradiation therapy is considered to be the core therapy for locally advanced NPC.

Though great progression has been made in NPC treatment, there are still over 20% patients developing into recurrence and metastasis. Epidermal growth factor receptor (EGFR) is a transmembrane receptor, and it is usually involved in the cellular proliferation, migration or invasion, and other cell biological activities [10].

Increasing evidence suggests that targeting EGFR might be a potential strategy for NPC therapy, in which EGFR is highly expressed in 85% of patients with advanced NPC [11]. To date, cetuximab and nimotuzumab are the monoclonal antibodies against EGFR tested in NPC clinical trials. Studies have attempted to evaluate the efficacy and toxicity of cetuximab combined with chemoradiation therapy in the treatment of advanced NPC, but the results have been inconformity [12–15].

Based on the above reasons, we performed this meta-analysis to evaluate the efficacy of concurrent radiocisplatin therapy with/without cetuximab from the aspects of curative rate and survival outcomes.

The article "Efficacy of Cetuximab in Nasopharyngeal Carcinoma Patients Receiving Concurrent Cisplatin-Radiotherapy: A Meta-Analysis" was retracted in 2023. Reasons: unreliable results or conclusions; concerns about the data; concerns about the peer review; concerns about the citations.

## 2. Methods

### 2.1. Literature Search Strategy

The databases including PubMed, Cochrane Library, EMBASE, China National Knowledge Infrastructure (CNKI), Wan Fang, and China Biology Medicine disc (CBM) were used to conduct literature searches (past to May 2022). Search terms included “cetuximab” and “radiotherapy” or “radiation therapy” and “cisplatin” or “cis-platinum” or “chemotherapy” and “nasopharyngeal carcinoma”.

### 2.2. Selection Criteria

The final included studies should meet the following criteria: (a) trials including patients that were diagnosed with nasopharyngeal carcinoma (NPC); (b) trials including patients who received both cetuximab and concurrent chemoradiotherapy, and the chemotherapy should use cisplatin; (c) trials reported as RCTs; and (d) the literature was published in English or Chinese, and the full text was available. When it comes to redundant publications, only the most recent studies were included. Studies belong to animal or cell experiments, case report, review, letter, and conference abstract, and those without full text were out of consideration. Besides, studies that were republished or irrelevant to the subject were excluded.

### 2.3. Data Extraction

The retrieved data were evaluated and screened independently by Lin Wang and Deyou Wei and were determined by Deyou Wei when it comes to disagreement. Studies in this meta-analysis included the following basic information: the name of first author, publication year and country, sample size, details of chemoradiotherapy, and outcomes (efficacy and survival).

### 2.4. Quality Assessment

The quality of the included trials was assessed by Newcastle-Ottawa Scale (NOS). Studies with a score above 6 are considered of high quality. All the 17 articles included in the current meta-analysis were deemed to be high-quality studies.

### 2.5. Statistical Analysis

All statistical analyses were performed using STATA 14.0 software (College Station, USA). For dichotomous data, relative risk (RR) and 95% confidence interval (CI) were reported. The *I*^2^ test was taken for heterogeneity between studies. If *I*^2^ ≤ 50% or *p* > 0.1, select the fixed-effects model; otherwise, select the random-effects model. Publication bias was evaluated through Begg's test and funnel plot, and *p* value less than 0.05 is considered significant.

## 3. Results

### 3.1. Study Characteristics

The literature selection process is shown in Figure 1. Initially, 763 studies were retrieved from the aforementioned databases based on the aim search terms, and 561 were left after removing duplicates. Next, 284 irrelevant studies were excluded by screening the titles or abstracts, and 75 were excluded due to ineligible data. Eventually, 17 trials were eligible for this meta-analysis. All of the 17 included studies were conducted in China, of which only 4 were published on SCI journals in English and the rest were published in Chinese journals (Table 1). In total, 2066 participants with NPC were involved in this meta-analysis. All the studies used cetuximab combined with chemoradiotherapy as observation group and chemoradiotherapy alone as the control. As for the outcomes, complete response (CR), partial response (PR), stable disease (SD), and progression disease (PD) were used to evaluate the treatment efficacy, and overall survival (OS), disease-free survival (DFS), metastasis-free survival (MFS), relapse-free survival (RFS), and progression-free survival (PFS) were used to assess the survival outcomes of the patients. NOS was used to evaluate the quality of the included literature. All 17 studies scored at least 6 and were considered high quality (Table 2).

The article "Efficacy of Cetuximab in Nasopharyngeal Carcinoma Patients Receiving Concurrent Cisplatin-Radiotherapy: A Meta-Analysis" was retracted in 2023. Reasons: unreliable results or conclusions; concerns about the data; concerns about the peer review; concerns about the citations.

### 3.2. Meta-Analysis

#### 3.2.1. Efficacy of Cetuximab Combined with Concurrent Chemoradiotherapy in NPC Treatment

Meta-analysis showed that cetuximab improved the therapy efficacy in NPC patients undergoing concurrent chemoradiotherapy. The CR, PR, SD, and PD data of the included studies were summarized in Table 3. As shown in Figure 2(a), the CR in patients who received the combined therapy of cetuximab and concurrent chemoradiotherapy was higher than those who only received concurrent chemoradiotherapy (RR = 1.92, 95% CI [1.61, 2.30], fixed-effects model), while no significant difference was noticed in PR (Figure 2(b)) between observation and control groups (RR = 0.96, 95% CI [0.80, 1.17], fixed-effects model). In addition, both SD and PD (Figures 2(c) and 2(d)) were lower in concurrent chemoradiotherapy with cetuximab than that without cetuximab (SD: RR = 0.67, 95% CI [0.51, 0.88], fixed-effects model; PD: RR = 0.24, 95% CI [0.15, 0.40], fixed-effects model). Furthermore, we calculated the objective response rate (ORR) and disease control rate (DCR) by the following formulae and conducted meta-analysis according to the calculated data. As shown in Figures 2(e) and 2(f), both ORR and DCR were higher in concurrent chemoradiotherapy with cetuximab than that without cetuximab (ORR: RR = 1.38, 95% CI [1.27, 1.51], fixed-effects model; DCR: RR = 1.12, 95% CI [1.05, 1.20], random-effects model).

(1) $$\begin{array}{c} \text{ORR}=\text{CR}+\text{PR},\\ \text{DCR}=\text{CR}+\text{PR}+\text{SD}. \end{array}$$

#### 3.2.2. Publication Bias of Treatment Efficacy

As shown in Figure 3, Begg's test was used to assess the potential publication bias. In general, funnel plots appeared symmetrical in CR, SD, PD, and DCR, and Begg's test results showed that no significant publication bias was in CR (*p* = 0.125), SD (*p* = 0.350), PD (*p* = 0.721), and DCR (*p* = 0.213). However, publication bias was noted in the meta-analysis of PR (*p* = 0.029) and ORR (*p* = 0.016).

The article "Efficacy of Cetuximab in Nasopharyngeal Carcinoma Patients Receiving Concurrent Cisplatin-Radiotherapy: A Meta-Analysis" was retracted in 2023. Reasons: unreliable results or conclusions; concerns about the data; concerns about the peer review; concerns about the citations.

#### 3.2.3. Survival Outcomes of NPC Patients Who Received Cetuximab Combined with Concurrent Chemoradiotherapy

The survival outcomes including OS, DFS, MFS, RFS, and PFS were summarized in Table 4. The results in our study show that cetuximab improved the survival outcomes of NPC patients. As shown in Figure 4(a), NPC patients who received cetuximab therapy had a higher OS than those who did not (RR = 1.10, 95% CI [1.02, 1.18], random-effects model). Likewise, cetuximab also improved DFS, MFS, and RFS in NPC patients undergoing concurrent chemoradiotherapy (Figures 4(b)–4(d), DFS: RR = 1.09, 95% CI [1.03, 1.15], fixed-effects model; MFS: RR = 1.06, 95% CI [1.01, 1.11], fixed-effects model; RFS: RR = 1.04, 95% CI [1.01, 1.07], fixed-effects model). However, as shown in Figure 4(e), there was no significance in PFS between NPC patients receiving cetuximab and those not receiving cetuximab (RR = 1.09, 95% CI [0.89, 1.32], random-effects model).

#### 3.2.4. Publication Bias of Survival Outcomes

Since only 2 studies provided DFS data and 3 offered PFS data, the publication bias towards these two outcomes was not conducted. As shown in Figure 5, funnel plots appeared symmetrical in OS, MFS, and RFS. The results of Begg's test showed that no significant publication bias was in these outcome indicators (OS: *p* = 0.060; MFS: *p* = 0.260; RFS: *p* = 1.000).

## 4. Discussion

NPC is a serious malignant tumor originating from nasopharyngeal epithelium. NPC has a unique geographical and ethnic distribution, and NPC is mostly found in East and Southeast Asians. NPC is the third most common carcinoma in southern China, with an incidence rate around 1/10,000 [31]. Currently, radiotherapy is still the main curative treatment for NPC, especially IMRT. NPC is likely to infiltrate in neighbour important tissues or organs, such as the brain stem, spinal cord, and optic chiasm. IMRT can target tumors at high doses while reducing doses to adjacent normal tissues [32]. Nevertheless, the 5-year survival rate of NPC patients with radiotherapy alone is only about 70% [33]. Thus, radiotherapy accompanied with concurrent or induction chemotherapy has been considered as a standard treatment.

Since cisplatin-based concomitant chemoradiotherapy may increase side effects in patients diagnosed with NPC; many other potential drugs in NPC treatment are under exploration. EGFR-based concomitant chemoradiation therapy is another novel alternative that may be suitable for advanced NPC treatment. Nowadays, monoclonal antibodies as well as small molecule tyrosine kinase inhibitors are used to against EGFR clinically. Cetuximab is one of the clinically used monoclonal antibodies. You et al. [20] demonstrated that concurrent chemoradiation therapy with cetuximab group exhibited better OS and DFS and distant metastasis-free survival (DMFS), while Li et al. [14] drew an opposite conclusion based on their case-control study. Due to the above paradoxes, we conducted this meta-analysis.

The article "Efficacy of Cetuximab in Nasopharyngeal Carcinoma Patients Receiving Concurrent Cisplatin-Radiotherapy: A Meta-Analysis" was retracted in 2023. Reasons: unreliable results or conclusions; concerns about the data; concerns about the peer review; concerns about the citations.

In total, 17 trials with 2066 patients were participated in this meta-analysis. The results in our study show that cetuximab improved the therapy efficacy in NPC patients who received concurrent cisplatin-radiotherapy. Cetuximab cotreatment improved the CR and reduced SD as well as PD. In addition, the survival outcomes were improved by cetuximab cotreatment including OS, DFS, MFS, and RFS. The heterogeneity in this study is not significant. We only found acceptable heterogeneity existing in the analyses of disease control rate (*I*^2^ = 50.4%, *p* = 0.028), overall survival (*I*^2^ = 50.9%, *p* = 0.032), and progression-free survival (*I*^2^ = 60.3%, *p* = 0.080).

However, the limitations of this study should be noted. First, all the included trials were conducted in China, and this may cause low study quality and regional disparity. Second, some of the included trials only provided limited data, which brings inaccuracy in subsequent meta-analysis including disease-free survival and progression-free survival. Last but not the least, publication bias was noticed in partial response and objective response rate. Nonetheless, this meta-analysis verified the positive efficacy of cetuximab in the combination of concurrent chemotherapy. It is recommended to include more high-quality studies for further evaluation.

## 5. Conclusions

To summarize, the results in this meta-analysis revealed that cetuximab could enhance the curative effects and improve the survival outcomes of NPC patients who received concurrent cisplatin-radiotherapy. All of the trials included were conducted in China, which may lead to low quality and regional disparity. Based on this, more trials with high quality are suggested for further assessment.

## Figures and Tables

**Figure 1:** Process of study selection.

**Figure 2:** Curative efficacy of cetuximab in NPC patients who received concurrent cisplatin-radiotherapy. Forest plots of (a) complete response, (b) partial response, (c) stable disease, (d) progression disease, (e) objective response rate, and (f) disease control rate.

The article "Efficacy of Cetuximab in Nasopharyngeal Carcinoma Patients Receiving Concurrent Cisplatin-Radiotherapy: A Meta-Analysis" was retracted in 2023. Reasons: unreliable results or conclusions; concerns about the data; concerns about the peer review; concerns about the citations.

**Figure 3:** Publication bias of curative efficacy. (a) Complete response. (b) Partial response. (c) Stable disease. (d) Progression disease. (e) Objective response rate. (f) Disease control rate.

**Figure 4:** Survival outcomes of cetuximab in NPC patients who received concurrent cisplatin-radiotherapy. Forest plots of (a) overall survival, (b) disease-free survival, (c) metastasis-free survival, (d) relapse-free survival, and (e) progression-free survival.

**Figure 5:** Publication bias of survival outcomes. (a) Overall survival. (b). Metastasis-free survival. (c) Relapse-free survival.

**Table 1:** Characteristics of the included studies.

First author	Year	Country	Sample size			Chemotherapy (cisplatin)	Radiotherapy (IMRT)	Cetuximab	Outcomes	
			T	E	C				Efficacy	Survival
P Yang^∗^ [16]	2021	China	126	63	63	80 mg/m^2^/3 w	66.0-75.9 Gy	400 mg/m^2^ loading dose and then 250 mg/m^2^/w	CR, PR, SD, and PD	OS, MFS, RFS, and PFS
J Liang [17]	2019	China	40	20	20	25 mg/m^2^, d_1_-d_3_/3 w	70 Gy	400 mg/m^2^ loading dose and then 250 mg/m^2^/w, 7 cycles	CR, PR	—
JJ Lu [18]	2018	China	64	32	32	20 mg/m^2^/3 w, 2 cycles	64-72 Gy	400 mg/m^2^ loading dose and then 250 mg/m^2^/w	CR, PR	—
WY Li [19]	2018	China	40	20	20	3 mg/m^2^, d_1_-d_3_/3 w	69 Gy	400 mg/m^2^ loading dose and then 250 mg/m^2^/w, 7 cycles	CR, PR, SD, and PD	OS
Y Li^∗^ [14]	2017	China	186	62	124	80-100 mg/m^2^/w, 2 cycles; 30-40 mg/m^2^/w, 5-7 cycles	68-76 Gy	400 mg/m^2^ loading dose and then 250 mg/m^2^/w, 6-7 cycles	—	OS, MFS, RFS, and PFS
WX Xia^∗^ [12]	2017	China	192	96	96	30-40 mg/m^2^/w; 80-100 mg/m^2^/3 w	Unclear dose	400 mg/m^2^ loading dose and then 250 mg/m^2^/w	—	OS, DFS, MFS, and RFS
R You^∗^ [20]	2017	China	791	102	689	10 mg/m^2^/3 w, 3 cycles	66-70 Gy	400 mg/m^2^ loading dose and then 250 mg/m^2^/w	—	OS, DFS, MFS, and RFS
ZY Yang [21]	2016	China	45	22	23	40 mg/m^2^/w, 6-8 cycles	73.96 Gy	400 mg/m^2^ loading dose and then 250 mg/m^2^/w, 7 cycles	CR, PR, SD, and PD	—
XX Wang [22]	2016	China	78	36	42	40 mg/m^2^/w, 6 cycles	66 Gy	40 mg/m^2^/w, 6 cycles	CR, PR, SD, and PD	OS, PFS
T Zeng [23]	2016	China	138	64	74	40 mg/m^2^/w, 6 cycles	76 Gy	400 mg/m^2^ loading dose and then 250 mg/m^2^/w, 6 cycles	CR, PR, SD, and PD	OS, MFS, and RFS
XQ Cao [24]	2016	China	40	20	20	33 mg/m^2^, d_1_-d_3_/3 w	69 Gy	400 mg/m^2^ loading dose and then 250 mg/m^2^/w, 7 cycles	CR, PR, SD, and PD	OS
ZQ Zhao [25]	2015	China	64	32	32	20 mg/m^2^/3 w, 4 cycles	64-72 Gy	400 mg/m^2^ loading dose and then 250 mg/m^2^/w	CR, PR, SD, and PD	—
MH Fu [26]	2015	China	64	36	28	20 mg/m^2^/4 w, 4 cycles	70 Gy	400 mg/m^2^ loading dose and then 250 mg/m^2^/w	CR, PR, SD, and PD	OS, MFS, and RFS
XL Fu [27]	2015	China	40	20	20	33 mg/m^2^, d_1_-d_3_/3 w	69 Gy	400 mg/m^2^ loading dose and then 250 mg/m^2^/w, 6 cycles	CR, PR, SD, and PD	OS
ZH Zheng [28]	2013	China	40	20	20	80 mg/m^2^/3 w, 2 cycles	69.96 Gy	400 mg/m^2^ loading dose and then 250 mg/m^2^/w, 7 cycles	CR, PR	—
CZ Wu [29]	2013	China	68	34	34	20 mg/m^2^, d_1_-d_4_/3 w, 2 cycles	64-68 Gy	100 mg/w, 7 cycles	CR, PR, SD, and PD	—
HY Ran [30]	2013	China	50	25	25	80 mg/m^2^/3 w, 2 cycles	70 Gy	400 mg/m^2^ loading dose and then 250 mg/m^2^/w	CR, PR, SD, and PD	—

T: total; E: experimental group; C: control group; CR: complete response; PR: partial response; SD: stable disease; PD: progression disease; OS: overall survival; DFS: disease-free survival; MFS: metastasis-free survival; RFS: relapse-free survival; PFS: progression-free survival. ^∗^Published on SCI journal in English.

The article "Efficacy of Cetuximab in Nasopharyngeal Carcinoma Patients Receiving Concurrent Cisplatin-Radiotherapy: A Meta-Analysis" was retracted in 2023. Reasons: unreliable results or conclusions; concerns about the data; concerns about the peer review; concerns about the citations.

**Table 2:** Methodological quality assessment of the included studies by Newcastle-Ottawa Scale.

Study	Selection				Comparability	Outcome			Total score
	Exposed cohort	Nonexposed cohort	Ascertainment of exposure	Outcome of interest		Assessment of outcome	Length of follow-up	Adequacy of follow-up	
P Yang	∗	∗	∗	∗	∗∗	∗	∗	∗	9
J Liang	∗	∗	∗	∗	∗	∗	—	—	6
JJ Lu	∗	∗	∗	∗	∗	∗	—	—	6
WY Li	∗	∗	∗	∗	∗	∗	∗	∗	8
Y Li	∗	∗	∗	∗	∗∗	∗	∗	—	8
WX Xia	∗	∗	∗	∗	∗∗	∗	∗	—	8
R You	∗	∗	∗	∗	∗	∗	∗	—	7
ZY Yang	∗	∗	∗	∗	∗	∗	—	—	6
XX Wang	∗	∗	∗	∗	∗∗	∗	∗	∗	9
T Zeng	∗	∗	∗	∗	∗∗	∗	∗	∗	9
XQ Cao	∗	∗	∗	∗	∗∗	∗	∗	∗	9
ZQ Zhao	∗	∗	∗	∗	∗	∗	—	—	6
MH Fu	∗	∗	∗	∗	∗∗	∗	∗	∗	9
XL Fu	∗	∗	∗	∗	∗∗	∗	∗	∗	9
ZH Zheng	∗	∗	∗	∗	∗∗	∗	—	—	7
CZ Wu	∗	∗	∗	∗	∗	∗	—	—	6
HY Ran	∗	∗	∗	∗	∗	∗	—	—	6

**Table 3:** Efficacy of cetuximab+concurrent cisplatin-radiotherapy.

Study	CR (%)		PR (%)		SD (%)		PD (%)	
	E	C	E	C	E	C	E	C
P Yang	50.8	31.7	39.7	41.3	9.5	15.9	0	11.1
J Liang	20.0	10.0	50.0	40.0	NA		NA	
JJ Lu	53.1	31.3	40.6	43.7	NA		NA	
WY Li	45.0	15.0	20.0	25.0	25.0	25.0	10.0	35.0
ZY Yang	50.0	17.4	36.4	34.8	9.1	34.8	4.5	13
XX Wang	80.6	61.9	13.9	16.7	5.6	19.1	0	2.4
T Zeng	40.6	13.5	31.3	29.7	21.9	32.4	6.2	24.4
XQ Cao	40.0	10.0	15.0	20.0	35.0	30.0	10.0	40.0
ZQ Zhao	34.4	21.9	43.8	31.3	18.8	21.9	3.1	25.0
MH Fu	36.1	14.3	30.6	28.6	22.2	32.1	5.6	25.0
XL Fu	10.0	5.0	40.0	25.0	40.0	55.0	10.0	15.0
ZH Zheng	75.0	25.0	15.0	45.0	NA		NA	
CZ Wu	52.9	26.5	20.6	32.4	17.6	14.7	8.8	26.5
HY Ran	68.0	44.0	28.0	32.0	4.0	24.0	0	0

E: experimental group; C: control group; CR: complete response; PR: partial response; SD: stable response; PD: progression disease; NA: not applicable.

**Table 4:** Survival of cetuximab+concurrent chemoradiotherapy.

Study	OS (%)		DFS (%)		MFS (%)		RFS (%)		PFS (%)	
	E	C	E	C	E	C	E	C	E	C
P Yang	84.1	79.4	NA		92.1	85.7	100	92.1	81	68.3
WY Li	40	20	NA		NA		NA		NA	
Y Li	90.3	91.1	NA		83.9	90.3	95.2	94.4	79	84.7
WX Xia	89.3	87.2	83.4	80.5	94.1	87.3	92.5	93.2	NA	
R You	96.6	92.9	93.5	86.9	94.6	89.3	97.8	94.7	NA	
XX Wang	88.9	69.1	NA		NA		NA		75	59.5
T Zeng	87.5	67.6	NA		78.1	64.9	87.5	81.1	NA	
XQ Cao	40	15	NA		NA		NA		NA	
MH Fu	88.9	67.9	NA		77.8	64.3	88.9	82.1	NA	
XL Fu	40	15	NA		NA		NA		NA	

E: experimental group; C: control group; OS: overall survival; DFS: disease-free survival; MFS: metastasis-free survival; RFS: relapse-free survival; PFS: progression-free survival.

The article "Efficacy of Cetuximab in Nasopharyngeal Carcinoma Patients Receiving Concurrent Cisplatin-Radiotherapy: A Meta-Analysis" was retracted in 2023. Reasons: unreliable results or conclusions; concerns about the data; concerns about the peer review; concerns about the citations.

## Data Availability

The labeled dataset used to support the findings of this study is available from the corresponding author upon request.
